The article "microRNA-98 inhibits the proliferation, invasion, migration and promotes apoptosis of breast cancer cells by binding to HMGA2" was retracted in 2021. Reasons: duplicated images; signs of a paper mill.

# microRNA-98 inhibits the proliferation, invasion, migration and promotes apoptosis of breast cancer cells by binding to HMGA2

**DOI:** 10.1042/BSR20180571

**Published:** 2018-09-19

**Authors:** Mi-Jia Wang, Hao Zhang, Jun Li, Hai-Dong Zhao

**Affiliations:** Department of Breast Surgery, The Second Affiliated Hospital of Dalian Medical University, Dalian 116000, P.R. China

**Keywords:** Breast cancer, High mobility group AT-hook 2, Invasion, microRNA-98, Migration, Proliferation

## Abstract

Breast cancer is a major contributor leading to cancer death in females worldwide. The aim of the present study was to investigate the effects of microRNA-98 (miR-98) on the processes of cell proliferation, invasion, migration and apoptosis by binding to high-mobility group AT-hook 2 (HMGA2) in breast cancer. Breast cancer tissues and adjacent normal tissues were collected from 112 patients suffering from breast cancer. The target relationship between miR-98 and HMGA2 was verified by in connection with the bioinformatics website as well as a dual-luciferase reporter assay, both of which provided evidence indicating that HMGA2 was a target gene of miR-98. Human breast cancer MDA-MB-231 cells were treated with miR-98 mimics, miR-98 inhibitors, siRNA-HMGA2 or miR-98 inhibitors + siRNA-HMGA2. 3-(4,5-Dimethylthiazol-2-yl)-2,5-diphenyltetrazolium bromide assay and flow cytometry methods were performed to determine cell proliferation, cell cycle and apoptosis, respectively, while a Transwell assay was employed to detect cell migration and invasion. Breast cancer tissues exhibited decreased miR-98 expression, while increased expression levels of HMGA2 were recorded. The mRNA and protein expressions of HMGA2, cell proliferation, cells at the S phase, cell migration, invasion, expressions of matrix metalloproteinase (MMP)2 as well as MMP9 were all reduced in response to miR-98 mimics or siRNA-HMGA2, while a contradictory trend was observed in the miR-98 inhibitors group. In conclusion, the results of the study demonstrate that miR-98 inhibits cell proliferation, migration and invasion, while acting to promote apoptosis by negatively regulating HMGA2 in breast cancer.

## Introduction

Driven by multiple genetic or epigenetic alterations and molecular events, breast cancer is a molecularly heterogeneous disease representing the most common type of cancer and a primary cause of mortality among women worldwide [1–3]. Breast cancer accounts for 12.2% of all tumor cases in Chinese women and 9.6% of all cancer-related deaths worldwide [4]. Certain nuclear receptors such as estrogen receptor-α and progesterone receptor have been reported to exhibit overexpressed levels in 70% of patients suffering from breast cancer [5]. In spite of the distinct progress in the clinical diagnosis, prognosis and treatment of breast cancer the survival rate of patients with metastatic breast cancer is still limited [6]. This is largely due to the complexity and poorly understood underlying cellular and molecular mechanisms associated with the occurrence of the disease. At present, most common therapeutic protocols for patients diagnosed with breast cancer include radical mastectomy, sentinel lymph node biopsy and systematic adjuvant treatment [7]. The effect of microRNA (miRNA) dysregulation on breast cancer has been extensively investigated since 2005, with certain miRNAs widely considered to play oncogenic roles in the occurrence and progression of breast cancer [8,9], while other miRNAs have been reported to play tumor-suppressing roles [10,11].

miRNAs belong to a family of small noncoding RNAs (19–25 nucleotide short RNAs) [12] that have been shown to control gene expression at a post-transcriptional level through the combination with complementary sequences at the 3′-untranslated regions (3′-UTR) of messenger RNAs (mRNAs) [13]. Furthermore, miRNAs have been reported to play a role in an array of biological processes, including cell proliferation, cell apoptosis and cell differentiation [14]. Reports have previously indicated that microRNA-98 (miR-98) is differentially expressed in the uterus of rats between the pre-receptive and receptive period [15]. Additionally, miR-98 has been shown to belong to the let-7 family, which represents a group of the most essential tumor suppressors that potentially contribute to the suppression of cell proliferation and cell invasion in cases of breast cancer [16,17]. Consistently, miR-98 expression has been reported to suppress the processes of angiogenesis as well as the survival, proliferation and metastasis of breast cancer cells by inhibiting the expressions of ALK4 as well as the matrix metalloproteinase (MMP)11 [18]. Moreover, the overexpression of miR-98 has been highlighted as a promising potential biomarker for patients with breast cancer [19]. The high-mobility group AT-hook 2 (HMGA2) is a target gene of miR-98, which has recently been discovered as a non-histone chromatin protein, sharing a close association with the development, invasion and metastasis of various types of cancers [20,21]. HMGA2 is overexpressed in breast cancer and has been shown to promote the invasion and metastasis of breast cancer [22,23]. Based on the exploration of literature as well as the current situation regarding the treatment of breast cancer, the central objective of the current study was to investigate whether miR-98 could suppress the cell proliferation, invasion and migration of breast cancer via binding to HMGA2 in a bid to discover a potential biomarker for improved breast cancer treatment.

## Materials and methods

### Ethics statement

The current study was conducted in strict accordance with the approval of the Ethics Committee of the Second Affiliated Hospital of Dalian Medical University. All participating patients signed informed consent documentation prior to enrollment into the study.

### Study subjects

Tumor specimens were collected from 112 patients who were previously pathologically diagnosed with breast cancer and received surgical treatment for the first time at the Second Affiliated Hospital of Dalian Medical University between August 2012 and June 2015. Patients were aged between 21 and 75 years old, with a median age of 51 years old. Among them, 55 patients were pre-menopausal. There were 36 cases at stage I, 53 cases at stage II and 23 cases at stage III [24]. The staging was based on the scores for nuclear pleomorphism, karyokinesis and glandular tube formation. The three parameters were scored on a system between 1 and 3 points. A lower score indicated a higher degree of differentiation, illustrating that the difference between breast cancer cells and normal breast cells was smaller. A total score of 8–9 points, 6–7 points and 3–5 points was regarded as stage III, stage II and stage I, respectively. All patients were diagnosed with breast cancer by means of tissue biopsy and pathological analyses. Pathological diagnosis criteria were in direct accordance with the ‘guideline and standard for the diagnosis and treatment of breast cancer in China (2007 edition)’ published by Chinese Anti-Cancer Association. The follow-up of patients lasted to June 2018. Both breast cancer tissues and adjacent normal tissues (5 cm away from tumor) were collected for the purposes of the present study.

### Immunohistochemistry

All tissues were fixed for 12 h with 4% paraformaldehyde, dehydrated, cleared, embedded in the paraffin and then sliced into sections. Paraffin-embedded sections were baked for 24–48 h at 60°C in an oven followed by dewaxing twice with xylene (10 min per time). After hydration in graded ethanol of 100%, 95%, 75% and 50% (5 min per time), the sections were rinsed with distilled water for 5 min and then washed with phosphate buffered saline (PBS) for 5 min. After the addition of one drop of hydrogen peroxide, the sections were incubated for 10 min at room temperature, followed by three PBS washes (3 min per wash). Antigen retrieval was conducted for 20 min in a microwave oven using citrate (pH = 6.0). The sections were then rinsed three times with PBS (3 min per wash) and incubated for 5 min at room temperature with one drop of normal goat serum. The serum was then subsequently discarded, and mouse anti-human HMGA2 primary antibody (ab184616, 1:1000, Abcam Inc., Cambridge, MA, U.S.A.) was added to incubate the sections at room temperature overnight. After three PBS washes (3 min per wash), the sections were incubated at room temperature for 15 min then added with 30 μl of biotin-labeled goat anti-mouse secondary antibody (ab6789, 1: 1000, Abcam Inc., Cambridge, MA, U.S.A.), followed by three additional PBS washes (3 min per time). Thereafter, the sections were further incubated with peroxidase-labeled streptavidin solution at room temperature for 15 min, followed by PBS three washes (3 min per time). Next, 3,3′-diaminobenzidine solution prepared in advance was used for chromogen, and the sample coloration was then observed for 3–5 min under a microscope. The sections were subsequently rinsed under running water and then counterstained with hematoxylin. After another round of washing with running water, the sections were dehydrated with 50%, 75%, 95% and 100% xylene and ethanol successively (5 min per time) and mounted with neutral resin. PBS was regarded as the negative control in replacement of the primary antibody. Brownish yellow granules in the cytoplasm were observed under a light microscope, and cells with brownish yellow granules were considered to represent positive expression cells. Five different views were randomly selected from each section. The number of positive expression cells was calculated under high power fields (×100), with the mean subsequently calculated. The positive expression levels were classified according to the percentage of tumor cells with positive expression in total tumor cells. Strong positive expression referred to a percentage >81%; positive expression referred to a percentage between 51% and 80%; weak positive expression referred to a percentage between 11% and 50%; negative expression referred to a percentage <10%.

### Reverse transcription quantitative polymerase chain reaction (RT-qPCR)

Breast cancer tissues (*n*=112) and adjacent normal tissues (*n*=112) were selected from clinically obtained specimens in order to conduct tissue experiments. The mRNA expression of miR-98 and HMGA2 among both sets of tissues was determined accordingly. The Trizol Reagent kit (Invitrogen, Carlsbad, CA, U.S.A.) was applied to extract the total RNA. Ultraviolet spectrophotometer and agarose gel electrophoresis were employed in order to detect RNA purity and concentration, and RNA integrity, respectively. Primescript RT reagent kit (Takara Biomedical Co., Ltd., Dalian, Liaoning, China) was applied for reverse transcription to prepare cDNA. Based on the kit instructions, reverse transcription conditions were set as follows: reverse transcription reaction at 37°C for 15 min and deactivation of reverse transcriptase at 85°C for 5 s. Primers of U6 (internal reference of miR-98), miR-98, β-actin and HMGA2 were designed, which were synthesized by Takara Biomedical Technology Co., Ltd. (Dalian, China) (Table 1). Reverse transcription quantitative polymerase chain reaction (RT-qPCR) experiment was conducted using the ABI7500 qPCR instrument (Applied Biosystems, Carlsbad, CA, U.S.A.). The reaction conditions were as follows: pre-denaturation at 95°C for 10 min, 40 cycles of denaturation at 95°C for 10 s, annealing at 60°C for 20 s and extension at 72°C for 34 s. The reaction system was comprised of: 2 μl of DNA template, 0.4 μl of PCR reverse primer (10 µM), 0.4 μl of PCR forward primer (10 µM), 10 μl of SYBR Premix Ex TaqTM II and 7.2 μl of sterile distilled water. U6 and β-actin considered as the internal references, and the 2^−ΔΔ*C*^_t_ method was applied to calculate the relative expression of target genes following the formula: ΔΔ*C*_t_ = [*C*_t_ (target gene) − *C*_t_ (reference gene)]_the experimental group_ − [*C*_t_ (target gene) − *C*_t_ (reference gene)]_the control group_. The experiment was repeated five times, with the aforementioned method also applicable for the subsequent cell experiments.

**Table 1:** Primer sequences for RT-qPCR

Gene	Prime sequence
U6	F: 5′-CTCGCTTCG GCAGCACA-3′
	R: 5′-AAC GCTTCACGA ATTTGCGT-3′
β-Actin	F: 5′-TGGACATCCGCAAAGAC-3′
	R: 5′-AGCACTGTGTTGGCGTACAG-3′
HMGA2	F: 5′-CAGCAGCAAGAACCAACCG-3′
	R: 5′-TGTTGTGGCCATTTCCTAGGT-3′
miR-98	F: 5′-GGGGTGAGGTAGTAAGTTGT-3′
	R: 5′-TGGGTGTCGTGGAGTC-3′

Note: F, forward; R, reverse.

### Western blot assay

Breast cancer tissues and adjacent normal tissues were cut into pieces, after which cell lysate was added to the tissues followed by a 30 min ice-bath. After high speed centrifugation, the supernatant was collected and bicinchoninic acid (Thermo Fisher Scientific Inc., Waltham, MA, U.S.A.) assay was used to detect the protein concentration. The samples were then adjusted to an equal concentration by lysate according to their respective concentration. After the loading buffer had been added, the samples were degenerated by heating in a water bath at 100°C for 5 min. Marker (Takara Biomedical Technology Co., Ltd., Dalian, China) and samples were added into sample wells of sodium dodecyl sulfate-polyacrylamide gel electrophoresis (SDS-PAGE) gel, with 60 μg/lane sample in 0.75 mm gel. Electrophoresis at 100 V was then conducted until the front of the Bromophenol Blue was observed to have reached the end of the gel. After SDS-PAGE separation, the proteins were transferred to polyvinylidene fluoride (PVDF) membranes (Merck Millipore, Billerica, MA, U.S.A.) at 100 V for 75 min by wet electrophoretic transfer means. Tris-buffered saline (TBS) buffer solution was employed for three PVDF membranes washes (5 min per wash), followed by blockade with 5% skim milk for 1 h. The membranes were then incubated with primary antibodies of rabbit anti HMGA2 (1:5000), MMP2 (1:100) and MMP9 (1:100), and diluted β-actin antibody (1: 200) (Bioss Biotechnology, Beijing, China) at 4°C overnight. After three TBS washes (5 min per wash), the membranes were placed into horseradish peroxidase-labeled goat anti-rabbit IgG (1: 2000, Cusabio Biotech Co., Ltd., Wuhan, China) and incubated for 1 h at room temperature. Finally, the membranes were rinsed three times with TBS (5 min per wash), and an electro-chemical luminescence (ECL) kit (GE Healthcare, Little Chalfont, Buckinghamshire, U.K.) was applied to reveal the Western blotting bands. β-Actin was regarded as the internal reference, while the marker protein utilized was purchased from Thermo Fisher Scientific Inc. (Waltham, MA, U.S.A.; #84785). The protein bands were analyzed by ImageJ2x software in order to determine the relative expressions of the different proteins. This method was also applied for the cell experiments.

### Dual-luciferase reporter assay

The bioinformatics website *microRNA.org* was employed in the process of identifying the relationship between miR-98 and HMGA2. 293T cell lines purchased from American Type Culture Collection (ATCC, Manassas, VA, U.S.A.) were incubated and sub-cultured at 37°C with 5% CO_2_ and saturated humidity with Dulbecco’s modified Eagle’s medium (DMEM) comprises 10% fetal bovine serum (FBS). Cells at the logarithmic growth phase were selected for further experimentation. The DNA of the adjacent normal breast cells was extracted based on instructions of TIAN amp Genomic DNA Kit (TIANGEN Biotech Co., Ltd., Beijing, China) in order to construct luciferase reporter vectors. Artificially synthesized HMGA2 3′-UTR segments were inserted into the pMIR-reporter plasmids through Spe I and Hind III cleavage sites. Next, the mutant sites of the complementary sequences were designed in wild-type (wt) HMGA2 (HMGA2-wt), digested by restriction enzyme and inserted into pMIR-reporter plasmids using T4 DNA ligase. The wt and mutant (mut) luciferase reporter plasmids with correct sequences were then confirmed by means of sequential analysis and then co-transfected with miR-98 into 293T cell lines, respectively. Dual-luciferase reporter assay system (E1910, Promega, Shanghai Haoran Biological Co., Ltd., Shanghai, China) was applied to detect luciferase activity. The former culture medium was discarded 48 h after transfection and the cells were then rinsed twice with PBS. The cells were then added with 100 μl of passive lysis buffer in each well and slightly shaken at room temperature for 15 min, followed by collection of the cell lysate. The program was set for 2 s for pre-reading and 10 s for value reading, with 100 μl of LARII Stop &Glo Reagent (Promega Corporation, Madison, WI, U.S.A.). added for each sampling session. Then, prepared LARII Stop &Glo Reagent (Promega Corporation, Madison, WI, U.S.A.) and luminescent plate or tube containing cell lysate (20 μl/per sample) were placed into a bioluminescence detector. Finally, the program was operated and data were recorded after fluorescence reading.

### Cell treatment

Human breast cancer cell line (MDA-MB-231) with high invasion and high migration was purchased from ATCC (Manassas, VA, U.S.A.). The cells were incubated in DMEM consisting of 8% FBS (Gibco Company, Grand Island, NY, U.S.A.) in an incubator at 37°C with 5% CO_2_. After sub-culture, third generation cells in the logarithmic growth phase were harvested for transfection purposes. Human breast cancer cells were classified into six groups, namely, the blank, negative control (NC), miR-98 mimics, miR-98 inhibitor, siRNA-HMGA2 and miR-98 inhibitors + siRNA-HMGA2 groups. miR-98 mimics and miR-98 inhibitors and their corresponding negative controls were all purchased from Invitrogen (Carlsbad, CA, U.S.A.), and siRNA-HMGA2 was synthesized by Shanghai GeneChem Limited Company (Shanghai, China). Cells in the logarithmic growth phase in each group were inoculated into a 6-well plate. When the cells had grown to 50% confluence, they were transfected in accordance with the instructions of the Lipofectamine 2000 kit (Invitrogen, Carlsbad, CA, U.S.A.). Next, 250 µl of serum-free Opti-MEM medium (Gibco Company, Grand Island, NY, U.S.A.) was applied to dilute 100 pmol miR-98 mimics, miR-98 inhibitors, siRNA-HMGA2, miR-98 inhibitors + siRNA-HMGA2 and negative controls (the final concentration was 50 nM). The mixtures were then slightly shaken and incubated for 5 min at room temperature. Next, 250 µl of serum-free Opti-MEM medium was used to dilute 5 µl of Lipofectamine 2000. After slight mixture, the mixtures were incubated at room temperature for 5 min. After full blending, the mixtures were incubated for 20 min at room temperature and added into culture wells. The cells were incubated at 37°C with 5% CO_2_, and the complete medium was replaced after 6–8 h. Further experiments were conducted 24–48 h after the cells were cultured.

### 3-(4,5-dimethylthiazol-2-yl)-2,5-diphenyltetrazolium bromide assay

The cells were collected and counted 48 h after transfection. After counting, cells (3 × 10^3^ to 6 × 10^3^ cells/well) were then inoculated into a 96-well plate with 200 μl of cells in each well. Six duplicated wells were set, and subsequent experiments were conducted at 0, 24, 48 and 72 h respectively: 20 μl of 3-(4,5-dimethylthiazol-2-yl)-2,5-diphenyltetrazolium bromide (MTT) solution (5 mg/ml) was added into each well, and then cells were incubated at 37°C for 4 h. After termination of the culturing process, the supernatant in wells was discarded. Thereafter, 150 μl of dimethyl sulfoxide was added into wells, and shaken for 10 min using enzyme-linked immunosorbent assay (Nanjing DeTie Laboratory Equipment Co., Ltd., Nanjing, Jiangsu, China). The optical density (OD) values in each well were measured at the wavelength of 570 nm. A cell growth curve was constructed with time as the abscissa and the OD value as the ordinate. The experiment was repeated three times.

### Flow cytometry

Cells, collected 48 h after cell transfection, were washed three times using PBS. The supernatant was subsequently discarded after centrifugation. The cells were then re-suspended by PBS and adjusted to a density of 1 × 10^5^ cells/ml. Subsequently, 1 ml of 75% ethanol pre-cooled at −20°C was used to fix cells at 4°C for 1 h, and the cells were then centrifuged at 7500 rpm for 5 min. The utilized cold ethanol was then discarded, and the cells were rinsed twice with PBS, followed by the removal of supernatant. Thereafter, cells were water bathed at 37°C under dark conditions for 30 min with 100 μl of RNase A and stained with propidium iodide (PI) (400 μl, Sigma Aldrich, St. Louis, MO, U.S.A.) at 4°C for 30 min under conditions void of light. A flow cytometry (FACScalibur, BD Biosciences, San Diego, CA, U.S.A.) was used to record red fluorescence at an excitation wavelength of 488 nm to detect cell cycle.

Forty-eight hours after transfection, THE cells were detached using ethylenediaminetetraacetic acid-free trypsin and collected into flow tubes in which the cells were centrifuged and supernatant was discarded. The cells were then washed three times with cold PBS and centrifuged again, with the supernatant discarded. Based on the fluorescein isothiocyanate (FITC)-labeled annexin V (Annexin-V-FITC) apoptosis detection kit (Sigma Aldrich, St. Louis, MO, U.S.A.), Annexin-V-FITC, PI and N-2-hydroxyethylpiperazine-N′-2-ethanesulfonic acid (HEPES) solutions (1:2:50) were mixed to prepare the Annexin-V-FITC/PI solution. Every 1 × 10^6^ cells were re-suspended in each 100 μl of Annexin-V-FITC/PI solution, shaken and mixed, followed by 15 min of incubation at room temperature and addition of 1 ml of HEPES solution with oscillation and mixing. Cell apoptosis analyses were conducted in connection with the detection of FITC and PI fluorescence at an excitation wavelength of 488 nm in a 525- and 620-nm bandpass filter.

### Transwell migration assay

Cells in each group were detached with trypsin 48 h after transfection and triturated repeatedly to prepare single cell suspension. The cells were then re-suspended with a serum-free medium after two PBS rinses, followed by adjustment of the cell concentration to 1.5 × 10^5^ cells/ml. Then, 100 μl of cell suspension was inoculated into the Transwell chamber, and 500 μl of culture medium with 10% FBS was added into the basolateral chamber. The chambers were removed 10–12 h after incubation at 37°C, with the cells that failed to penetrate through the membrane rubbed away using a cotton bud. The cells were then fixed with 95% ethanol for 15 min and stained by 0.1% Crystal Violet for 10 min. After three PBS rinses and natural air-drying, the chambers were inverted on a glass slide and photographed using the up-right fluorescence microscope. Five views (200×) were randomly selected from each filter membrane to count the number of transmembrane cells. The experiment was repeated five times.

### Transwell invasion assay

Serum-free medium was applied to dilute the Matrigel (1: 7), and then 50 μl of diluted Matrigel was inoculated into each chamber. The prepared chambers were all placed in an incubator at 37°C for 4 h for following experiments. Trypsin was used to detach the cells in each group 48 h after transfection, once the cells were confirmed to have dissociated into a single cell suspension through repeated trituration. After two PBS rinses, the cells were re-suspended using a serum-free medium, with the cell concentration then adjusted to 1.5 × 10^5^ cells/ml. Next, 100 μl of cell suspension was inoculated into the apical chamber covered by diluted Matrigel, while 500 μl of culture medium with 10% FBS was added to the basolateral chamber. The chambers were removed 10–12 h after incubation at 37°C, and cells that failed to penetrate through the membrane in chamber were rubbed away using a cotton bud. The cells were then fixed with 95% ethanol for 15 min and stained by 0.1% Crystal Violet for 10 min. After three PBS rinses and natural air-drying, the chambers were inverted on glass slides and photographed using the up-right fluorescence microscope. Five views (200×) were randomly selected from each filter membrane to count the number of transmembrane cells. The experiment was repeated five times.

### Statistical analysis

The SPSS 21.0 statistical software (IBM Corp. Armonk, NY, U.S.A.) was used to analyze all experimental data. Measurement data were presented as the mean ± standard deviation. Comparisons among multiple groups were analyzed by one-way analysis of variance, while comparisons between two groups were analyzed by *t*-test. A value of *P*<0.05 was indicative of statistical significance.

## Results

### Positive expression rate of HMGA2 is higher in the breast cancer tissues

Immunohistochemical staining was performed in order to determine the positive expression rate of HMGA2 protein among the breast cancer tissues as well as the adjacent normal tissues (*n*=112). The results illustrated that the protein expression of HMGA2 was predominantly located in the cytoplasm (Figure 1A). The positive expression of HMGA2 was represented by a brownish yellow staining. The HMGA2 expression was strongly positive in the breast cancer tissues. The results provided verification that the positive expression rate of HMGA2 was significantly elevated in the breast cancer tissues in comparison with the adjacent normal tissues (*P*<0.05, Figure 1B).

**Figure 1:** Immunohistochemical staining demonstrates that positive expression rate of HMGA2 is higher in the breast cancer tissues (**A**) Immunohistochemical staining of HMGA2 in breast cancer tissues and adjacent normal tissues (×200). (**B**) Comparison of the positive expression rate of HMGA2 between breast cancer tissues and adjacent normal tissues; *P<0.05 versus the adjacent normal tissues. Sample: breast cancer tissues (*n*=112) and adjacent normal tissues (*n*=112).

### Low expression of miR-98 along with high expression of HMGA2 in the breast cancer tissues

RT-qPCR and Western blot assay methods were performed in order to determine the expressions of miR-98 and HMGA2 among the breast cancer tissues and adjacent normal tissues (*n*=112). RT-qPCR results (Figure 2A) indicated that the expression of miR-98 was evidently lower in the breast cancer tissues at I (*n*=36), II (*n*=53) or III (*n*=23) stages when compared with the adjacent normal tissues (*P*<0.05), while the HMGA2 mRNA expression exhibited a contrasting trend (*P*<0.05). No significant difference was observed regarding the expression of miR-98 and mRNA expression of HMGA2 between the breast cancer tissues at the I stage and those at the II stage (*P*>0.05); notable differences among the breast cancer tissues at the III stage in comparison with that of those at the I and II stages were detected (*P*<0.05). Western blot assay (Figure 2B,C) suggested that the breast cancer tissues possessed a significantly higher HMGA2 protein expression than that of the adjacent normal tissues, with higher stages reflective of more significant difference (*P*<0.05). The data obtained provided evidence proving that miR-98 is lowly expressed with high expressions of HMGA2 in breast cancer tissues. More importantly, the 112 cases of breast cancer patients were classified into high expression group and low expression group, with the median value of miR-98 expression as a cut-off value. The results indicated that the patients in the high expression group of miR-98 showed higher overall survival rate than those in the low expression group of miR-98.

**Figure 2:** Low expressions of miR-98 along with high expressions of HMGA2 in the breast cancer tissues, determined by RT-qPCR and Western blot assay (**A**) miR-98 expression and mRNA expression of HMGA2 in breast cancer tissues at I, II and III stages and adjacent normal tissues detected by RT-qPCR. (**B**) Protein bands of HMGA2 protein expression in breast cancer tissues and adjacent normal tissues. (**C**) Quantitative analysis of HMGA2 protein expression in breast cancer tissues and adjacent normal tissues. (**D**) Low expression of miR-98 exerted adverse effects on the survival of breast cancer patients. The median cut-off value was determined by RT-qPCR; *P<0.05 versus the adjacent normal tissues. Sample size: breast cancer tissues (*n*=112) and adjacent normal tissues (*n*=112); breast cancer tissues at I stage (*n*=36), breast cancer tissues at II stage (*n*=53) and breast cancer tissues at III stage (*n*=23).

### HMGA2 is a target gene of miR-98

Furthermore, we examined whether miR-98 could directly regulate HMGA2 by means of target prediction program and luciferase activity determination. The bioinformatics website *microRNA.org* (http://www.microrna.org/microrna/home.do) revealed there to be specific binding sites of miR-98 to 3′-UTR of HMGA2, suggesting miR-98 could bind to HMGA2 in a targeted manner (Figure 3A). The results of the dual-luciferase reporter assay verified that in the miR-98 mimics group, the luciferase activity of cells co-transfected with Wt-miR-98/HMGA2 plasmid were notably reduced when compared with the NC group (*P*<0.05); however among those co-transfected with mut-miR-98/HMGA2 plasmid no significant difference was detected in regard to the luciferase activity in comparison with the NC group (*P*<0.05) (Figure 3B). The results indicated that miR-98 could specifically bind to HMGA2.

**Figure 3:** HMGA2 is a target gene of miR-98, confirmed by bioinformatics website and dual-luciferase reporter assay (**A**) Bioinformatics website predicted that miR-98 targets HMGA2. (**B**) Dual-luciferase reporter assay verifies that miR-98 targets HMGA2; *P<0.05 versus the NC group.

### miR-98 is a negative regulator of HMGA2

RT-qPCR was performed to determine the expression of miR-98 and mRNA expression of HMGA2 after cell transfection in order to ascertain as to whether miR-98 could influence the mRNA expression of HMGA2. As illustrated by Figure 4A, compared with the NC and blank groups, the miR-98 mimics group presented significantly higher levels of miR-98 expression (*P*<0.05), the miR-98 inhibitors and miR-98 inhibitors + siRNA-HMGA2 groups had significantly lower miR-98 expression (both *P*<0.05), while no significant difference was observed in the siRNA-HMGA2 group (all *P*<0.05). Compared with the NC and blank groups, HMGA2 mRNA expression was down-regulated in the miR-98 mimics and siRNA-HMGA2 groups but up-regulated in the miR-98 inhibitors group (all *P*<0.05), no significant difference in relation to the HMGA2 mRNA expression was detected between the miR-98 mimics and siRNA-HMGA2 groups (*P*<0.05). Moreover, no significant difference was observed in terms of the HMGA2 mRNA expression in the miR-98 inhibitors + siRNA-HMGA2 group between the NC and blank groups (all *P*<0.05).

**Figure 4:** miR-98 negatively regulates mRNA and protein expression of HMGA2, determined by RT-qPCR and Western blot assay (**A**) miR-98 expression and mRNA expression of HMGA2 in human breast cancer MDA-MB-231 cells after transfection, determined by RT-qPCR. (**B**) Protein bands of HMGA2 protein expression in human breast cancer MDA-MB-231 cells after transfection, determined by Western blot assay. (**C**) Quantitative analysis of HMGA2 protein expression in human breast cancer MDA-MB-231 cells after transfection, determined by Western blot assay; *P<0.05 versus the blank and NC groups; NC, negative control.

In addition, a Western blot assay was conducted in order to determine the protein expression of miR-98 and HMGA2 after cell transfection in order to verify whether miR-98 could influence the protein expressions of HMGA2. The results of the Western blot assay (Figure 4B,C) revealed that compared with the NC and blank groups, the HMGA2 protein expression in the miR-98 mimics and siRNA-HMGA2 groups was significantly decreased after transfection (all *P*<0.05), while no significant difference in relation to the HMGA2 protein expression in the miR-98 mimics and siRNA-HMGA2 groups was detected (*P*<0.05). Besides, the miR-98 inhibitors group had significantly higher HMGA2 protein expression (all *P*<0.05) compared with the blank and NC groups. No statistical significant difference was observed regarding the HMGA2 protein expression between the miR-98 inhibitors + siRNA-HMGA2, blank and NC groups (*P*<0.05).

Taken together, based on the results obtained, we concluded that miR-98 could negatively regulate the mRNA and protein expression of HMGA2.

### Up-regulated miR-98 expression or down-regulated HMGA2 expression inhibits breast cancer cell proliferation

MTT assay was applied in order to construct cell growth curves. The OD values are depicted in Figure 5. Compared with the blank and NC groups, cell proliferation in breast cancer was inhibited in the miR-98 mimics and siRNA-HMGA2 groups (all *P*<0.05), while enhanced levels were observed in the miR-98 inhibitors group (*P*<0.05). No significant difference was detected in the miR-98 inhibitors + siRNA-HMGA2 group in terms of cell proliferation between the blank and NC groups (all *P*<0.05). These results demonstrated that overexpressed miR-98 could suppress the proliferation of breast cancer cells, while up-regulated HMGA2 expression could promote cell proliferation.

**Figure 5:** Up-regulated miR-98 expression or down-regulated HMGA2 expression inhibits breast cancer cell proliferation, detected by MTT assay *P<0.05 versus the blank and NC groups.

### miR-98 inhibits cell cycle entry and induces apoptosis of breast cancer cells by inhibiting HMGA2

An investigation was conducted to identify the effect of miR-98 on the cell cycle distribution of breast cancer cells by means of PI single staining (Figure 6A,B). Fewer cells at the S phase and inhibited cell proliferation were detected in the miR-98 mimics and siRNA-HMGA2 groups. Compared with the blank and NC groups, the miR-98 mimics and siRNA-HMGA2 groups displayed more cells at the G1 phase and less cells at the S phase (all *P*<0.05), while a contrasting result was observed in the miR-98 inhibitors group (all *P*<0.05). There was no significant difference in relation to the proportion of cells at the G1 and S phases between the miR-98 inhibitors + siRNA-HMGA2, blank and NC groups (all *P*<0.05). These results proved that overexpressed miR-98 inhibited the cell progression into the S phase, as well as indicating that miR-98 could suppress cell proliferation by inhibiting HMGA2.

**Figure 6:** miR-98 represses breast cancer cell cycle entry and induces breast cancer cell apoptosis by inhibiting HMGA2, detected by flow cytometry (**A**) Cell cycle detected by flow cytometry. (**B**) Comparisons of cell cycle distribution among seven groups. (**C**) Apoptosis of breast cancer cells in the scatter plots of flow cytometry. (**D**) Apoptosis rate of breast cancer cells in each group; *P<0.05 versus the blank and NC groups; NC, negative control.

Annexin V/PI double staining was performed to detect breast cancer cell apoptosis after cell transfection, as illustrated in Figure 6C,D. The results demonstrated that 4 h after transfection, the cell apoptosis rates in the blank, NC, miR-98 mimics, miR-98 inhibitors, siRNA-HMGA2 and miR-98 inhibitors + siRNA-HMGA2 groups were (27.745 ± 7.745)%, (26.182 ± 6.182)%, (43.291 ± 3.291)%, (13.99 ± 3.99)%, (41.715 ± 1.715)%, (28.715 ± 8.715)% respectively. Compared with the blank and NC groups, the cell apoptosis in the miR-98 mimics and siRNA-HMGA2 groups was significantly higher, while that of the miR-98 inhibitors group was lower (all *P*<0.05). No significant difference was detected in the miR-98 inhibitors + siRNA-HMGA2 group in terms of cell apoptosis when compared with the blank and NC groups (all *P*<0.05). These findings illustrated that miR-98 could induce cell apoptosis by inhibiting HMGA2.

### miR-98 inhibits breast cancer cell migration and invasion by suppressing HMGA2

The effects of miR-98 on breast cancer cell migration and invasion were explored using Transwell assays. Figure 7A,B revealed that compared with the blank and NC groups, cell migration was inhibited in the miR-98 mimics and siRNA-HMGA2 groups (both *P*<0.05), but was elevated in the miR-98 inhibitors group (*P*<0.05). No significant difference in terms of cell migration was found among the miR-98 inhibitors + siRNA-HMGA2, blank and NC groups (all *P*<0.05). Figure 7C,D illustrates the comparison between the blank and NC groups, demonstrating that cell invasion was suppressed in the miR-98 mimics and siRNA-HMGA2 groups (both *P*<0.05), while displaying enhanced levels in the miR-98 inhibitors group (*P*<0.05). No significant difference was observed in the miR-98 inhibitors + siRNA-HMGA2 group in terms of cell invasion when compared with that of the blank and NC groups (all *P*<0.05).

**Figure 7:** miR-98 inhibits breast cancer cell migration and invasion by suppressing HMGA2 by Transwell assays (**A**) Cell migration in human breast cancer MDA-MB-231 cells by Transwell migration assay. (**B**) The number of migrating human breast cancer MDA-MB-231 cells in each group. (**C**) Cell invasion in human breast cancer MDA-MB-231 cells by Transwell invasion assay. (**D**) The number of invasive human breast cancer MDA-MB-231 cells in each group. (**E**) Protein bands of expressions of migration and invasion related proteins (MMP2 and MMP9) in human breast cancer MDA-MB-231 cells after transfection. (**F**) Quantitative analysis of protein expressions of migration and invasion related proteins (MMP2 and MMP9) in human breast cancer MDA-MB-231 cells after transfection; *P<0.05 versus the blank and NC groups.

In order to further verify the effects of miR-98 on breast cancer cell migration and invasion, a Western blot assay was performed, depicted in Figure 7E,F. Compared with the blank and NC groups, the protein expressions of MMP2 and MMP9 were down-regulated in the miR-98 mimics and siRNA-HMGA2 groups (both *P*<0.05), while up-regulated levels were observed in contrast in the miR-98 inhibitors group (*P*<0.05). No significant difference was detected in the miR-98 inhibitors + siRNA-HMGA2 group in terms of the protein expressions of MMP2 and MMP9 when compared with the blank and NC groups (all *P*<0.05).

Therefore, it was concluded that miR-98 could inhibit breast cancer cell migration and invasion by suppressing HMGA2.

## Discussion

As a molecularly heterogeneous disease, breast cancer continues to be a major clinical stumbling block, representing a leading reason of cancer deaths worldwide [2,3]. Reports have recently indicated that both miR-98 and HMGA2 regulate breast cancer cell proliferation, invasion and survival [18,23]. Notably, miR-98 has been shown to target HMGA2 [20]. Hence, the present study set out to investigate the role of miR-98 in modulating cell proliferation, invasion, migration and apoptosis of breast cancer by regulating HMGA2, in an attempt to identify a novel target for the treatment of breast cancer.

Our study illustrated among breast cancer cells there to be low expressions of miR-98 expression and high mRNA and protein expression of HMGA2. HMGA2 was determined to be a direct target gene of the miR-98. Previous reports have provided verification that miR-98, which is part of the let-7 family, is a negative regulator for HMGA2 oncogene expression [25]. Zhao et al. [19] suggested there to be an association between dysregulated miR-98/let-7 and breast cancer, which has been further indicated in other studies to be a common event in patients with breast cancer, highlighting the potential of miR-98/let-7 as a novel biomarker for breast cancer treatment. In this study, we also provided evidence that patients with high expression of miR-98 showed higher overall survival rate than those with low expression of miR-98. Numerous reports have documented distinctly descended miR-98 expression in certain solid tumors, such as the head and neck squamous cell carcinoma and nasopharyngeal carcinoma [21,26]. Moreover, miR-98 expression was down-regulated after the treatment of chemokine (C-C motif) ligand 18 (CCL18) in MCF-7 and MDA-MB-231 breast cancer cells [17]. High expression of HMGA2 has been found in breast cancer, which was largely consistent with the findings of our study [23]. Similarly, HMGA2 expression in breast cancer patients has been reported to be correlated with metastasis and poor prognoses [21]. Yun et al. [27] demonstrated that the epigenetic regulator HMGA2 was targeted by let-7, which again was consistent with the findings of the current study. Similarly, Chen et al. [20] reported that miR-98 was negatively associated with HMGA2 in tumor tissues, as well as suggesting that miR-98 could directly target HMGA2, lending further support to our results.

In addition, it was observed in the current study that overexpressed miR-98 could inhibit breast cancer cell proliferation, cell invasion and cell migration, while acting to facilitate cell apoptosis by negatively targeting HMGA2. The expressions of the proteins related to the processes of migration and invasion, including MMP2 and MMP9, exhibited markedly decreased levels in breast cancer cells. Various reports have highlighted the significant role played by miRNAs in the processes of cell proliferation, apoptosis and differentiation, while overexpressed miR-98 has been previously proven to inhibit hepatocellular carcinoma cell proliferation, migration and invasion [15,28]. More specifically, Lin et al*.* [17] verified that the tumor suppressor, let-7/miR-98, suppresses breast cancer cell proliferation, invasion and migration, consistent with our study. Reports have revealed that in cases of prostate cancer, down-regulated HMGA2 may significantly suppress cell proliferation, migration and invasion but elevate cell apoptosis. Both breast cancer and prostate cancer are often analyzed together; reduced HMGA2, targeted by miR-98, has been speculated to possibly inhibit breast cancer cell proliferation, migration, invasion and promote cell apoptosis [29,30]. Sun et al*.* [23] demonstrated that inhibited HMGA2 suppressed the invasion and metastasis of breast tumor cells, which was shown to be beneficial to the survival of breast cancer patients, indicating that the negative targeting of HMGA2 by miR-98 could inhibit cell invasion and metastasis in breast cancer. Additionally, the expression of MMPs which function as tumor suppressors has been correlated with the processes of invasion and metastasis [31]. Moreover, miR-98 expression has been speculated to inhibit breast cancer cell proliferation, invasion, survival and angiogenesis through the reduction of MMP11 expression, which was a finding parallel to our study [18]. Shi et al. [29] revealed that HMGA2 silencing depressed expressions of MMPs, which were related to cell invasion and migration. HMGA2 has been reported to decrease the expressions of MMP2 and MMP9 [32].

## Conclusions

In conclusion, our study revealed there to be low expressions of miR-98 and high expressions of HMGA2 among breast cancer cells, in addition to discovering that miR-98 directly targets HMGA2. Overexpressed miR-98 was found to suppress breast cancer cell proliferation, invasion and migration, while acting to promote cell apoptosis by negatively regulating HMGA2. However, the sample size is limited and the finer mechanism by which miR-98 and negatively regulated HMGA2 inhibits breast cancer cell proliferation, invasion, migration, invasion as well as the promotion of cell apoptosis requires further investigation, which may help identify a novel treatment target for breast cancer.

## Abbreviations

HMGA2: high-mobility group AT-hook 2
MMP: matrix metalloproteinase
RT-qPCR: reverse transcription quantitative polymerase chain reaction

## References

[1] ZhangJ., LiuD., FengZ., MaoJ., ZhangC., LuY. (2016) MicroRNA-138 modulates metastasis and emt in breast cancer cells by targeting vimentin. Biomed. Pharmacother., 77, 135–141, 10.1016/j.biopha.2015.12.01826796277

[2] MichailidouK., HallP., Gonzalez-NeiraA., GhoussainiM., DennisJ., MilneR.L. (2013) Large-scale genotyping identifies 41 new loci associated with breast cancer risk. Nat. Genet. 45, 353–361, 361e351-352 10.1038/ng.2563 23535729PMC3771688

[3] KaoJ., SalariK., BocanegraM., ChoiY.L., GirardL., GandhiJ. (2009) Molecular profiling of breast cancer cell lines defines relevant tumor models and provides a resource for cancer gene discovery. PLoS One 4, e6146 10.1371/journal.pone.0006146 19582160PMC2702084

[4] FanL., Strasser-WeipplK., LiJ.J., St LouisJ., FinkelsteinD.M., YuK.D. (2014) Breast cancer in China. Lancet Oncol. 15, e279–e289 10.1016/S1470-2045(13)70567-9 24872111

[5] LuM., DingK., ZhangG., YinM., YaoG., TianH. (2015) MicroRNA-320a sensitizes tamoxifen-resistant breast cancer cells to tamoxifen by targeting ARPP-19 and ERRgamma. Sci. Rep. 5, 8735 10.1038/srep08735 25736597PMC4348640

[6] LuoM. and GuanJ.L. (2010) Focal adhesion kinase: a prominent determinant in breast cancer initiation, progression and metastasis. Cancer Lett. 289, 127–139 10.1016/j.canlet.2009.07.005 19643531PMC2854647

[7] LeeJ., ParkS., KimS., KimJ., RyuJ., ParkH.S. (2015) Characteristics and survival of breast cancer patients with multiple synchronous or metachronous primary cancers. Yonsei Med. J. 56, 1213–1220 10.3349/ymj.2015.56.5.1213 26256962PMC4541649

[8] KumarS., KeerthanaR., PazhanimuthuA. and PerumalP. (2013) Overexpression of circulating miRNA-21 and miRNA-146a in plasma samples of breast cancer patients. Indian J. Biochem. Biophys. 50, 210–214 23898484

[9] LiuH., WangY., LiX., ZhangY.J., LiJ., ZhengY.Q. (2013) Expression and regulatory function of miRNA-182 in triple-negative breast cancer cells through its targeting of profilin 1. Tumour Biol. 34, 1713–1722 10.1007/s13277-013-0708-0 23430586

[10] LiJ., KongX., ZhangJ., LuoQ., LiX. and FangL. (2013) MiRNA-26b inhibits proliferation by targeting PTGS2 in breast cancer. Cancer Cell Int. 13, 7 10.1186/1475-2867-13-7 23374284PMC3599806

[11] ShahN.R. and ChenH. (2014) MicroRNAs in pathogenesis of breast cancer: implications in diagnosis and treatment. World J. Clin. Oncol. 5, 48–60 10.5306/wjco.v5.i2.48 24829851PMC4014796

[12] LuK., WangJ., SongY., ZhaoS., LiuH., TangD. (2015) miRNA-24-3p promotes cell proliferation and inhibits apoptosis in human breast cancer by targeting p27Kip1. Oncol. Rep. 34, 995–1002 10.3892/or.2015.4025 26044523

[13] BaerC., ClausR. and PlassC. (2013) Genome-wide epigenetic regulation of miRNAs in cancer. Cancer Res. 73, 473–477 10.1158/0008-5472.CAN-12-3731 23316035

[14] BelverL., PapavasiliouF.N. and RamiroA.R. (2011) MicroRNA control of lymphocyte differentiation and function. Curr. Opin. Immunol. 23, 368–373 10.1016/j.coi.2011.02.001 21353514PMC3109091

[15] XiaH.F., JinX.H., CaoZ.F., ShiT. and MaX. (2014) MiR-98 is involved in rat embryo implantation by targeting Bcl-xl. FEBS Lett. 588, 574–583 10.1016/j.febslet.2013.12.026 24444606

[16] YangY., AgoT., ZhaiP., AbdellatifM. and SadoshimaJ. (2011) Thioredoxin 1 negatively regulates angiotensin II-induced cardiac hypertrophy through upregulation of miR-98/let-7. Circ. Res. 108, 305–313 10.1161/CIRCRESAHA.110.228437 21183740PMC3249645

[17] LinX., ChenL., YaoY., ZhaoR., CuiX., ChenJ. (2015) CCL18-mediated down-regulation of miR98 and miR27b promotes breast cancer metastasis. Oncotarget 6, 20485–20499 2624487110.18632/oncotarget.4107PMC4653020

[18] SiragamV., RutnamZ.J., YangW., FangL., LuoL., YangX. (2012) MicroRNA miR-98 inhibits tumor angiogenesis and invasion by targeting activin receptor-like kinase-4 and matrix metalloproteinase-11. Oncotarget 3, 1370–1385 10.18632/oncotarget.717 23211491PMC3717799

[19] DengZ.Q., YinJ.Y., TangQ., LiuF.Q., QianJ., LinJ. (2014) Over-expression of miR-98 in FFPE tissues might serve as a valuable source for biomarker discovery in breast cancer patients. Int. J. Clin. Exp. Pathol. 7, 1166–1171 24696733PMC3971322

[20] ChenZ., ChengQ., MaZ., XiH., PengR. and JiangB. (2013) Overexpression of RKIP inhibits cell invasion in glioma cell lines through upregulation of miR-98. Biomed. Res. Int. 2013, 695179 10.1155/2013/695179 24392454PMC3874320

[21] HebertC., NorrisK., ScheperM.A., NikitakisN. and SaukJ.J. (2007) High mobility group A2 is a target for miRNA-98 in head and neck squamous cell carcinoma. Mol. Cancer 6, 5 10.1186/1476-4598-6-5 17222355PMC1783857

[22] WendP., RunkeS., WendK., AnchondoB., YesayanM., JardonM. (2013) WNT10B/beta-catenin signalling induces HMGA2 and proliferation in metastatic triple-negative breast cancer. EMBO Mol. Med. 5, 264–279 10.1002/emmm.201201320 23307470PMC3569642

[23] SunM., SongC.X., HuangH., FrankenbergerC.A., SankarasharmaD., GomesS. (2013) HMGA2/TET1/HOXA9 signaling pathway regulates breast cancer growth and metastasis. Proc. Natl. Acad. Sci. U.S.A. 110, 9920–9925 10.1073/pnas.130517211023716660PMC3683728

[24] FarhatG.N., WalkerR., BuistD.S., OnegaT. and KerlikowskeK. (2010) Changes in invasive breast cancer and ductal carcinoma in situ rates in relation to the decline in hormone therapy use. J. Clin. Oncol. 28, 5140–5146 10.1200/JCO.2010.29.5121 21060026PMC3020688

[25] XiangQ., TangH., YuJ., YinJ., YangX. and LeiX. (2013) MicroRNA-98 sensitizes cisplatin-resistant human lung adenocarcinoma cells by up-regulation of HMGA2. Pharmazie 68, 274–281 23700794

[26] AlajezN.M., ShiW., HuiA.B., BruceJ., LenarduzziM., ItoE. (2010) Enhancer of Zeste homolog 2 (EZH2) is overexpressed in recurrent nasopharyngeal carcinoma and is regulated by miR-26a, miR-101, and miR-98. Cell Death Dis. 1, e85 10.1038/cddis.2010.64 21368858PMC3035896

[27] YunJ., FrankenbergerC.A., KuoW.L., BoelensM.C., EvesE.M., ChengN. (2011) Signalling pathway for RKIP and Let-7 regulates and predicts metastatic breast cancer. EMBO J. 30, 4500–4514 10.1038/emboj.2011.312 21873975PMC3230370

[28] WangC.Y., ZhangJ.J., HuaL., YaoK.H., ChenJ.T. and RenX.Q. (2016) MicroRNA-98 suppresses cell proliferation, migration and invasion by targeting collagen triple helix repeat containing 1 in hepatocellular carcinoma. Mol. Med. Rep. 13, 2639–2644 10.3892/mmr.2016.4833 26846175

[29] ShiZ., WuD., TangR., LiX., ChenR., XueS. (2016) Silencing of HMGA2 promotes apoptosis and inhibits migration and invasion of prostate cancer cells. J. Biosci. 41, 229–236 10.1007/s12038-016-9603-3 27240983

[30] SaadF., AdachiJ.D., BrownJ.P., CanningL.A., GelmonK.A., JosseR.G. (2008) Cancer treatment-induced bone loss in breast and prostate cancer. J. Clin. Oncol. 26, 5465–5476 10.1200/JCO.2008.18.4184 18955443

[31] HillionJ., WoodL.J., MukherjeeM., BhattacharyaR., Di CelloF., KowalskiJ. (2009) Upregulation of MMP-2 by HMGA1 promotes transformation in undifferentiated, large-cell lung cancer. Mol. Cancer Res. 7, 1803–1812 10.1158/1541-7786.MCR-08-0336 19903768PMC3069640

[32] YanJ., ZhangY., ShiW., RenC., LiuY. and PanY. (2016) The critical role of HMGA2 in regulation of EMT in epithelial ovarian carcinomas. Tumour Biol. 37, 823–828 10.1007/s13277-015-3852-x 26250458

